# Intra- and Interrater Agreement of Face Esthetic Analysis in 3D Face Images

This article has been retracted.

**DOI:** 10.1155/2023/3717442

**Published:** 2023-04-10

**Authors:** Minsoo Park, Hang-Nga Mai, Mai Yen Mai, Thaw Thaw Win, Du-Hyeong Lee, Cheong-Hee Lee

**Affiliations:** ^1^Department of Prosthodontics, School of Dentistry, Kyungpook National University, 2177 Dalgubeoldae-ro, Jung-Gu, Daegu 41940, Republic of Korea; ^2^Dental School of Hanoi University of Business and Technology, 10000 Hanoi, Vietnam; ^3^Institute for Translational Research in Dentistry, Kyungpook National University, 2177 Dalgubeoldae-ro, Jung-Gu, Daegu 41940, Republic of Korea

## Abstract

The use of three-dimensional (3D) facial scans for facial analysis is increasing in maxillofacial treatment. The aim of this study was to investigate the consistency of two-dimensional (2D) and 3D facial analyses performed by multiple raters. Six men and four women (25–36-year-old) participated in this study. The 2D images of the smiling and resting faces in the frontal and sagittal planes were obtained. The 3D facial and intraoral scans were merged to generate virtual 3D faces. Ten clinicians performed facial analyses by investigating 14 indices of 2D and 3D faces. Intra- and interrater agreements of the results of 2D and 3D facial analyses within and among the participants were evaluated. The intrarater agreement between the 2D and 3D facial analyses varied according to the indices. The highest and lowest agreements were found for the dental crowding index (0.94) and smile line curvature index (0.56) in the frontal plane, and Angle's classification (canine) index (0.98) and occlusal plane angle index (0.55) in the profile plane. In the frontal plane, the interrater agreements were generally higher for the 3D images than for the 2D images, while in the profile plane, the interrater agreements were high in the Angle's classification (canine) index however low in the other indices. Several occlusion-related indices were missing in the 2D images because the posterior teeth were not observed. Esthetic analysis results between 2D and 3D face images can differ according to the evaluation indices. The use of 3D faces is recommended over 2D images to increase the reliability of facial analyses, as it can fully assess both esthetic and occlusion-related indices.

## 1. Introduction

A symmetrical face, along with an attractive smile, is essential for maintaining and improving a person's esthetic appearance, self-esteem, and quality of life [1]. Therefore, to enhance treatment quality, facial esthetic analysis has been performed as a routine diagnostic method in various dental fields such as orthodontics, prosthetics, and maxillofacial surgery [2]. Face analysis is performed to evaluate the structure of a face using various esthetic indicators [3]. This analysis provides valuable data to effectively plan the treatment, enable direct consultations with the patient, and help predict the prognosis of treatment [4]. Therefore, a visualized treatment plan can be established through the results of the analysis and consultations for clinicians to effectively communicate with the patient and finalize the goal of treatment.

In the past, esthetic analysis primarily consisted of two-dimensional (2D) radiographs and camera photographs [5]. Panoramic radiographs and lateral cephalometry were used to perform skeletal analysis [6], and soft tissues were analyzed in a static state using camera photographs [7]. With these static images, various methods were suggested to analyze the face for ideal beauty. For the simple and intuitive comparison, evaluation of the facial symmetry, and the proportion of each facial part using the golden ratio has been considered the most fundamental method [8, 9]. Moreover, growth analysis, such as the Ricketts, Downs, and Steiner methods, and computational analysis by Pascal are conducted [2, 10]. However, in this 2D analysis, image distortion and related errors can occur. For instance, 2D radiographic techniques, such as panoramic and lateral cephalometry, lack transverse information and the precise location of anatomical structures [11]. In addition, 2D profile photographs may not completely reflect actual facial perceptions because facial depth and shape are not considered [3]. As traditional 2D images cannot exactly reflect real three-dimensional (3D) results, communication between dentists and patients becomes challenging.

With the advancement of digital dentistry, devices, and computer software for facial esthetic analysis have been developed [12, 13]. Currently, 3D reconstruction of the jaws using cone-beam computed tomography is widely used for radiographic diagnosis in dental treatments [14]. The 3D soft tissue data on the face can also be obtained using 3D face scanning [15]. To obtain the structure of the oral cavity, intraoral optical scanning is currently replacing conventional physical impressions and stone-cast fabrication [16]. When extraoral and intraoral data are acquired digitally, it becomes possible to produce a virtual face in 3D. Although 3D facial analysis has attracted significant interest, there have been only a few studies on the reproducibility of 3D analysis. Therefore, we aimed to compare the consistency of the 3D-face-based facial esthetic analysis conducted by multiple evaluators with that of conventional 2D-photographic-based facial analysis.

## 2. Materials and Methods

To collect images for facial analysis, 10 adults (six men, four women; 25–36 years of age) with no history of facial injury, pathology, or cosmetic/maxillofacial surgery were recruited. The participants provided consent and were aware of the purpose of the study. The study procedure is shown in Figure 1 and was approved by the ethical research board of Kyungpook National University Dental Hospital (approval number: KNUDH-2021-11-05-00).

For data collection, 2D facial images of all participants were obtained using a digital camera (D5600, Nikon, Tokyo, Japan) with a macro lens (AF-S Dx Micro Nikkor 85 mm 1 : 3,5G ED VR, Nikon,, Tokyo, Japan) (Figures 2(a) and 2(b)). Frontal and sagittal-plane photographs of the smiling and resting faces were taken. The distance between the camera and the participant was set at 2 m, and the head position was maintained with the Frankfort plane parallel to the floor. Smile photographs were obtained pronouncing “cheese” sounds to make participants smile consistently. To eliminate the impact caused by the change of light source, all photographs were taken in the same place indoors with led lights. All photos were taken with the setting of aperture of f/11, shutter speed of 1/60s, and standard ISO speeds 200. Photographs were saved in the joint photographic expert's group (JPEG) format with a resolution of 3000 dots per inch (DPI). The 3D facial images were collected using a 3D facial scanner (RAYFace; Ray, Seoul, Korea) (Figure 2(c) and 2(d)). The 3D images were acquired of smiling and resting faces with and without an extraoral marker tray [17]. The dental arch was scanned using an intraoral scanner (i700, MEDIT, Seoul, Korea) to acquire images of the dentition, which were saved in the polygon file format. In image management software (RAYFace), the 3D facial and intraoral scan images were merged using the extraoral marker tray images (Figure 3). All 2D and 3D image collections were performed by a trained clinician

Facial esthetic analysis was performed by investigating 14 indices (Table 1). Among these, eight indices were evaluated in the frontal images, and six indices were evaluated in the profile image (Figure 4). Ten clinicians participated in the esthetic analysis. Before initiating the analysis, the evaluators were educated regarding the definition and evaluation methods of each esthetic index. All evaluations were performed in images without a built-in measurement tool. The degrees of intrarater agreement between the results of 2D and 3D esthetic facial analyses in the same participant and interrater agreement among the evaluators on the results of 2D and 3D esthetic facial analyses were evaluated.

## 3. Results

In the facial esthetic evaluation at the frontal plane, the degree of intrarater agreement between 2D and 3D face image analyses was the highest for the dental crowding index (0.94) and the lowest for the smile line curvature index (0.56) (Table 2). Overall, the interpupillary line, midline deviation, and dental crowding indices showed high interrater agreement, while the smile line curvature, lip line level, and facial type indices demonstrated low interrater agreement values (Table 3). The interrater agreement in the commissural line and facial symmetry indices was higher in the 3D images than in the 2D images; meanwhile, the degree of agreement in midline deviation and lip line level indices was lower in 3D images than in 2D images.

Regarding facial esthetic evaluation at the profile plane, the intrarater agreement of results between 2D and 3D face image analyses was the highest in the Angle's classification (canine) index (0.98) and the lowest in the occlusal plane angle index (0.55) (Table 4). The interrater agreement was high for Angle's classification index; however, for the other indices, the agreement values were generally low (Table 5). There were missing values in the evaluation of the 2D images for occlusal plane angle and Angle's classification indices. In particular, Angle's classification index, which is based on the relationship with the first molar, could not be examined by a single evaluator in the 2D images. For all indices of the profile images, the interrater agreements in the 3D images were similar to those in the 2D images.

## 4. Discussion

This study was designed to investigate the consistency between 2D and 3D facial analyses and to examine the degree of agreement among ratters. The results of this study showed that the intrarater agreement of the results between 2D and 3D face image analyses differed according to the evaluation indices. For example, an intrarater agreement between 2D and 3D face images was high for Angle's classification (canine) index, whereas it was low for the occlusal plane angle index. Therefore, it is thought that different face analyses can be made in the same evaluator according to the image the decision was made.

In the frontal plane evaluations, the indices with a high interrater agreement in both 2D and 3D images were the interpupillary line, midline deviation, dental crowding, and Angle's classification indices, because these esthetic indices are easy to observe and less affected by the angle of viewing the image and have objective judgement criteria. As for the profile plane evaluations, Angle's classification index demonstrated high intra- and interrater agreement because it was evaluated according to a fixed reference point: the buccal groove of the mandibular first molar and mesiobuccal cusp of the maxillary first molar. Meanwhile, the smile line curvature, lip line level, facial type, profile shape, Frankfort-mandibular plane angle, and lip protrusion indices showed a low interrater agreement. The inconsistency of judgements may arise from the subjective characteristics of the criteria because the observers' perspectives could be different, depending on the viewing angle [18]. In this study, the interrater agreement was low for most indices that used reference planes such as the occlusal, Camper's, mandibular, and Frankfort planes evaluated in the profile plane. As these planes are imagined, intuitive evaluation of these planes without directly observing them on an image may be less objective [19]. In esthetic evaluations, subjective judgments may occur, which may cause differences in judgments between ratters [20]. Therefore, rather than the type of image, the precise definition of the index for facial analysis and the evaluation method that can be performed objectively are considered important.

In 2D facial images, Angle's classification of molars was not evaluated. This was because the molars could not be observed in the 2D facial profile photographs. The 3D imaging technologies have been used in dentistry [21]. Currently, the facial and intraoral scan images can be merged to generate a complete virtual 3D face with a full dental arch. Furthermore, polygonal resources such as tooth and jaw models can be managed using 3D computer image software; thus, the state of the dentition can be evaluated by adjusting the transparency of the facial scan image and clinicians can also obtain an in-depth perception of both the teeth and face by freely changing the angle of view [22]. Accordingly, the 3D method enabled occlusion-related evaluations, which were impossible using the 2D method. Furthermore, 3D image presentation can aid in measuring the actual sizes and shapes of anatomical structures [23]. Thus, 3D environmental settings may facilitate treatment planning and virtual treatment practices [24, 25].

The accuracy of the image integration of the digital dental model and the 3D facial image is affected by the capability of the 3D face scans to provide a clear appearance of the anterior teeth [26]. In the photogrammetry face scanning method, multiple single-lens reflex cameras are positioned at a fixed distance and angle from the object to ensure overlapping fields of view; thus, the oral area image in the face scan is often deformed because of limitations in the depth recognition of device and light accessibility. The faulty image reconstruction of the tooth structure on the face scan could be problematic for the tooth-based matching method to correctly conduct the dentofacial image integrations [17]. In this study, to enhance the accuracy of image matching, an extraoral marker tray was used. The artificial markers supply distinct reference landmarks that appeared in both the oral and facial images; thereby facilitating the image-matching process and enhancing the accuracy of the matching results.

This study attempted to include the effects of human-related factors by involving multiple participants and raters; however, the sample size was limited. Considering the diversity of ethnicity and clinical experience, large-scale clinical studies are required to generalize the findings of this study [27]. Additionally, the use of only a single 3D face scanner could be another limitation of this study. Previous studies reported that ambient spectral light could influence the quality of images in the scanners with stereophotogrammetry, but had little impact in the scanners with laser and structured-light technologies [28, 29]. During 3D image taking, direct and strong ambient light may cause a glare effect that obscures the surface details [28]. Thus, further studies should include various types of 3D face scanners and computer software for 3D visualization with various light sources.

## 5. Conclusions

Within the limitations of this study, the following conclusions were drawn:

1. Based on the agreement ratio of the 2D and 3D facial analyses, the facial analysis results within and among the evaluators could be different according to the evaluation indices and type of facial images
2. Esthetic indices that are less affected by the angle of viewing the image and have objective judgment criteria exhibited higher interrater agreement in both 2D and 3D images. Thus, to increase the reliability of the facial analysis, objective assessment criteria, and evaluation methods are needed
3. The use of 3D faces combined with tooth images is recommended over 2D images, as it enables both esthetic and occlusion-related evaluations, which were not allowed in the 2D method

## Figures and Tables

**Figure 1:** Workflow of this study.

**Figure 2:** Face image collection. (a) Two-dimensional (2D) photograph at the frontal plane. (b) 2D photograph at the sagittal plane. (c) Three-dimensional (3D) scan image at the frontal plane. (d) 3D scan image at the sagittal plane.

**Figure 3:** Facial scan with an extraoral marker tray.

**Figure 4:** Evaluation index for facial esthetic analysis. (a) Frontal image. (b) Profile image. (A) Interpupillary line. (B) Commissural line. (C) Smile line curvature. (D) Midline deviation. (E) High lip line. (F) Dental crowding. (G) Facial type. (H) Facial symmetry. (I) Occlusal plane angle. (J) Angle's classification (canine). (K) Angle's classification (first molar). (L) Profile shape. (M) Frankfort-mandibular plane angle (FMA). (N) Lip protrusion.

**Table 1:** Evaluation index for facial esthetic analysis.

View	Facial expression	Evaluation index	Level
Frontal	Smile	Interpupillary line	Parallel Rt. slanted Lt. Slanted
		Commissural line	Parallel Rt. slanted Lt. Slanted
		Smile line curvature	Upward Straight Downward
		Midline deviation	Accompany Rt. Lt.
		High lip line	High Intermediate Low
		Dental crowding	Crowding Normal Spacing
	Resting	Facial type	Dolichocephalic Mesocephalic Brachycephalic
		Facial symmetry	Symmetrical Asymmetrical

Profile	Smile	Occlusal plane angle	Parallel Clockwise Counter clockwise
		Angle's classification (canine)	I II III
		Angle's classification (first molar)	I II III
	Resting	Profile shape	Normal Convex Concave
		Frankfort-mandibular plane angle (FMA)	High Average Low
		Lip protrusion	Protruded Intermediate Retruded

**Table 2:** Intrarater agreement of evaluation results between the two-dimensional (2D) and three-dimensional (3D) frontal face images.

Evaluation index	Image	*N*	AR (%)
Interpupillary line	2D-3D	100	88
Commissural line	2D-3D	100	74
Smile line curvature	2D-3D	100	56
Midline deviation	2D-3D	100	82
Lip line level	2D-3D	100	74
Dental crowding	2D-3D	100	94
Facial type	2D-3D	100	78
Facial symmetry	2D-3D	100	82

AR: agreement ratio; 2D-3D: between 2D and 3D images.

**Table 3:** Interrater agreement of evaluation results in the two-dimensional (2D) and three-dimensional (3D) frontal face images.

Evaluation index	Image	*N*	AR (%)
Interpupillary line	2D	100	94
	3D	100	86
Commissural line	2D	100	70
	3D	100	82
Smile line curvature	2D	100	59
	3D	100	54
Midline deviation	2D	100	91
	3D	100	81
Lip line level	2D	100	71
	3D	100	59
Dental crowding	2D	100	96
	3D	100	94
Facial type	2D	100	62
	3D	100	62
Facial symmetry	2D	100	79
	3D	100	87

AR: Agreement ratio.

**Table 4:** Intrarater agreement of evaluation results between the two-dimensional (2D) and three-dimensional (3D) profile face images.

Evaluation index	Image	N	AR (%)
Occlusal plane angle	2D-3D	93	0.55
Angle's classification (canine)	2D-3D	49	0.98
Angle's classification (1st molar)	2D-3D	0	—
Profile shape	2D-3D	100	0.73
Frankfort-mandibular plane angle	2D-3D	100	0.63
Lip protrusion	2D-3D	100	0.64

AR: Agreement ratio, 2D-3D: Between 2D and 3D images.

**Table 5:** Interrater agreement of evaluation results in the two-dimensional (2D) and three-dimensional (3D) profile face images.

Evaluation index	Image	*N*	AR (%)
Occlusal plane angle	2D	93	59
	3D	100	64
Angle's classification (canine)	2D	49	98
	3D	100	88
Angle's classification (1st molar)	2D	0	—
	3D	100	81
Profile shape	2D	100	57
	3D	100	58
Frankfort-mandibular plane angle	2D	100	60
	3D	100	63
Lip protrusion	2D	100	53
	3D	100	51

AR: agreement ratio.

## Data Availability

The data used to support the findings of this study have been included in this manuscript.

## References

[1] Moskowitz M. E., Nayyar A. (1995). Determinants of dental esthetics: a rational for smile analysis and treatment. *Compendium of Continuing Education in Dentistry*.

[2] Margossian P., Laborde G., Koubi S., Tardivo D., Magne P. (2021). Determination of facial references for esthetic restorative treatment. *The International Journal of Periodontics & Restorative Dentistry*.

[3] Sarver D. M., Ackerman M. B. (2003). Dynamic smile visualization and quantification: part 2. Smile analysis and treatment strategies. *American Journal of Orthodontics and Dentofacial Orthopedics*.

[4] Benecke M., Kasper J., Heesen C., Schäffler N., Reissmann D. R. (2020). Patient autonomy in dentistry: demonstrating the role for shared decision making. *BMC Medical Informatics and Decision Making*.

[5] Rifkin R. (2000). Facial analysis: a comprehensive approach to treatment planning in aesthetic dentistry. *Practical Periodontics and Aesthetic Dentistry*.

[6] Akcam M. O., Altiok T., Ozdiler E. (2003). Panoramic radiographs: a tool for investigating skeletal pattern. *American Journal of Orthodontics and Dentofacial Orthopedics*.

[7] Ayaz I., Shaheen E., Aly M. (2020). Accuracy and reliability of 2-dimensional photography versus 3-dimensional soft tissue imaging. *Imaging Science in Dentistry*.

[8] Prokopakis E. P., Vlastos I. M., Picavet V. A. (2013). The golden ratio in facial symmetry. *Rhinology*.

[9] Rossetti A., De Menezes M., Rosati R., Ferrario V. F., Sforza C. (2013). The role of the golden proportion in the evaluation of facial esthetics. *The Angle Orthodontist*.

[10] Magne P., Salem P., Magne M. (2018). Influence of symmetry and balance on visual perception of a white female smile. *The Journal of Prosthetic Dentistry*.

[11] Harris D., Horner K., Gröndahl K. (2012). E.A.O. Guidelines for the use of diagnostic imaging in implant dentistry 2011. A consensus workshop organized by the European Association for Osseointegration at the Medical University of Warsaw. *Clinical Oral Implants Research*.

[12] Marques D., Alves R., Pinto R., Caramês J., Francisco H., Caramês J. (2021). Facial scanner accuracy with different superimposition methods: an in vivo study. *The International Journal of Prosthodontics*.

[13] Mai H. N., Lee D. H. (2020). Accuracy of Mobile device-compatible 3D scanners for facial digitization: systematic review and meta-analysis. *Journal of Medical Internet Research*.

[14] Kaasalainen T., Ekholm M., Siiskonen T., Kortesniemi M. (2021). Dental cone beam CT: an updated review. *Physica Medica*.

[15] Li Z., Giunta R. E., Frank K., Schenck T. L., Koban K. C. (2022). Reproducibility of novel soft-tissue landmarks on three-dimensional human facial scan images in Caucasian and Asian. *Aesthetic Plastic Surgery*.

[16] Mangano F., Gandolfi A., Luongo G., Logozzo S. (2017). Intraoral scanners in dentistry: a review of the current literature. *BMC Oral Health*.

[17] Mai H. N., Lee D. H. (2022). Effects of artificial extraoral markers on accuracy of three-dimensional dentofacial image integration: smartphone face scan versus stereophotogrammetry. *Journal of Personalized Medicine*.

[18] Rotundo R., Nieri M., Bonaccini D. (2015). The smile esthetic index (SEI): a method to measure the esthetics of the smile. An intra-rater and inter-rater agreement study. *European Journal of Oral Implantology*.

[19] Čelar A., Tafaj E., Graf A., Lettner S. (2018). Association of anterior and posterior occlusal planes with different angle and skeletal classes in permanent dentitions : a lateral cephalometric radiograph study. *Journal of Orofacial Orthopedics*.

[20] Cosyn J., Thoma D. S., Hämmerle C. H., De Bruyn H. (2017). Esthetic assessments in implant dentistry: objective and subjective criteria for clinicians and patients. *Periodontology 2000*.

[21] Kapila S. D., Nervina J. M. (2015). CBCT in orthodontics: assessment of treatment outcomes and indications for its use. *Dento Maxillo Facial Radiology*.

[22] Rao A., Tait I., Alijani A. (2015). Systematic review and meta-analysis of the role of mental training in the acquisition of technical skills in surgery. *American Journal of Surgery*.

[23] de Vos B. D., Wolterink J. M., de Jong P. A., Leiner T., Viergever M. A., Isgum I. (2017). ConvNet-based localization of anatomical structures in 3-D medical images. *IEEE Transactions on Medical Imaging*.

[24] Piedra-Cascón W., Fountain J., Att W., Revilla-León M. (2021). 2D and 3D patient's representation of simulated restorative esthetic outcomes using different computer-aided design software programs. *Journal of Esthetic and Restorative Dentistry*.

[25] Urbankova A. (2010). Impact of computerized dental simulation training on preclinical operative dentistry examination scores. *Journal of Dental Education*.

[26] Mai H.-N., Lee D.-H. (2021). The effect of perioral scan and artificial skin markers on the accuracy of virtual dentofacial integration: stereophotogrammetry versus smartphone three-dimensional face-scanning. *International Journal of Environmental Research and Public Health*.

[27] Rokaya D., Suttagul K., Sapkota B., Maharjan S. K. (2018). Gender based comparison of the relationships of maxillary anterior teeth and facial measurements. *Journal of International Dental and Medical Research*.

[28] Flynn M. J., Badano A. (1999). Image quality degradation by light scattering in display devices. *Journal of Digital Imaging*.

[29] Thongma-Eng P., Amornvit P., Silthampitag P., Rokaya D., Pisitanusorn A. (2022). Effect of ambient lights on the accuracy of a 3-dimensional optical scanner for face scans: an in vitro study. *Journal of Healthcare Engineering*.

